This article has been retracted.

# Porous Lactose as a Novel Ingredient Carrier for the Improvement of Quercetin Solubility *In Vitro*

**DOI:** 10.1155/2021/2586990

**Published:** 2021-08-27

**Authors:** Wen Liu, Tong-Tong Wang, Xiao-Luan Tang, Fei-Ya Jiang, Xiao Yan, Jun Deng

**Affiliations:** ^1^Department of Pharmacy, Hunan Provincial People's Hospital (The First-affiliated Hospital of Hunan Normal University), Changsha 410005, China; ^2^Hunan Provincial Key Laboratory of Emergency and Critical Care Metabonomics, Changsha 410005, China; ^3^Department of Pharmacy, Medical School of Hunan Normal University, Changsha 410013, China; ^4^Department of Pharmacy, Fujian Health College, Fuzhou 350101, China

## Abstract

In this work, quercetin was loaded in the highly-porous lactose via the adsorption of quercetin molecules in ethanol. The method aims to improve the quercetin solubility and the loading capacity of lactose. The method relates to the synthesis of the highly-porous lactose with a particle size of ∼35 *μ*m, a mean pore width of ∼30 nm, a BET surface area of 35.0561 ± 0.4613 m^2^/g, and a BJH pore volume of ∼0.075346 cc/g. After the quercetin loading in ethanol, BET surface area and BJH pore volume of porous lactose were reduced to 28.8735 ± 0.3526 m^2^/g and 0.073315 cc/g, respectively. The reduction rate was based on the quercetin loading efficiency of highly-porous lactose. DSC analysis and XRD analysis suggest that the sediments of quercetin in the nanopores of porous lactose are crystalline. FTIR spectroscopy results suggest that there is no significant interaction between quercetin and lactose. The highly-porous lactose had a higher loading efficiency of 20.3% (w/w) compared to the *α*-lactose (with 5.2% w/w). The release rates of quercetin from the highly-porous lactose tablets were faster compared to the conventional *α*-lactose carrier.

## 1. Introduction

Quercetin, a member of flavonoid family, is present in vegetables, grains, and fruits and is one of the most prominent dietary antioxidants [1]. Due to the number and location of free hydroxyl groups in quercetin molecule, its antioxidant activity is higher than that of the well-known antioxidant molecules ascorbic acid and rutin (Figure 1) [2, 3]. In addition to its antioxidant activity, quercetin has a series of pharmacological activities, including antiviral [4], antibacterial [5], anti-inflammatory [6], anticancer [7], and antihypertensive [8]. However, the low water solubility, low bioavailability, and poor chemical stability of quercetin restrict its clinical application, which is related to the poor crystallinity and solubility [9, 10].

In order to overcome these shortcomings of quercetin and make it play a better role in clinical practice, many technologies have been adopted to improve the oral bioavailability of quercetin. Among them, the better method is nanocarrier drug delivery system, which is a research hotspot in the field of pharmacy in recent years [11]. Hatahet et al. suspended quercetin (5%) in 0.5% aqueous solution of polyoxymethylene sorbitol monooleate and ground it for 5 minutes to obtain quercetin nanosuspension. The results showed that the saturated solubility and dissolution of quercetin nanosuspension were 7.56 times and 6 times of those of raw materials, respectively [12]. Sun et al. prepared quercetin-polylactic acid nanoparticles by emulsion-solvent evaporation method. Compared with quercetin suspension, the relative bioavailability of quercetin nanoparticles was 525.07% [13]. Therefore, it is very important to adopt various pharmaceutical methods to improve the solubility and bioavailability of hydrophobic drugs.

Lactose is one of the most widely used excipients in oral pharmaceutical preparations because of its wide sources, low cost, high solubility, stable physical and chemical properties, and low hygroscopicity [14, 15]. However, lactose has poor porosity and surface area, which limits its application as drug carrier [16,17]. Previous studies have shown that porous lactose has high porosity and surface area, which can improve drug loading and drug solubility [18, 19]. Spray drying and antisolvent technology are two main methods to prepare porous lactose [20]. In our work, we chose the antisolvent method to prepare porous lactose to load the hydrophobic drug quercetin, so as to improve the drug loading and drug solubility.

## 2. Materials and Methods

### 2.1. Materials

*α*-Lactose monohydrate (≥90%) was of pharmaceutical grade and purchased from Jiangsu Dawning Pharmaceutical Co., Ltd., China. Dimethyl sulfoxide (DMSO, >99%), ethanol (>99.9%), and HCl were of AR grade and purchased from Shanghai Aladdin Biochemical Technology Co., Ltd., China. Quercetin (purity >96%) was purchased from Shanghai Sarn Chemical Technology Co., Ltd., China.

### 2.2. Methods

#### 2.2.1. Antisolvent Precipitation for Preparation of Porous Lactose

Porous lactose was prepared by antisolvent method. Dimethyl sulfoxide was used to dissolve lactose, and ethanol was used as antisolvent to precipitate lactose. 1 microgram of *α*-lactose monohydrate was dissolved in 0.5 ml of dimethyl sulfoxide. Then, it was added into 10 ml of ethanol, it was shook properly and let to stand for 1 hour. After stabilization, lactose was centrifuged at 4000 rpm and then dried to constant weight by blowing N_2_ gas.

#### 2.2.2. Preparation of Quercetin Loaded Lactose for Tableting

Quercetin was loaded in lactose by physical adsorption. We dissolved 50 mg quercetin in ethanol to obtain quercetin solution and added 2 ml quercetin solution to 0.3 g *α*-lactose and porous lactose prepared as mentioned above with pipette. After standing for half an hour to fully absorb the load, we centrifuged to remove the supernatant, blow dried, and blew N_2_ gas for a constant weight. The quercetin-lactose tableting was performed with a tabletop tableting machine (Tianjin Tianguang FW-4, China) equipped with a tableting die (diameter: 8.0 mm).

### 2.3. Determination of Drug Loading Efficiency and *In Vitro* Dissolution Test

The drug content of lactose was determined by UV-vis spectrophotometer (Cary 60). The maximum absorption wavelength (*λ*max) of quercetin in solution was observed at 384 nm by using the ultraviolet scanning function from 200 nm to 800 nm. Calibration curves were generated for quantitative measurement to determine drug loading and release. As for the dissolution test, we prepared tablets at 37 °C in 500 ml of dissolution medium 0.1 N hydrochloric acid buffer pH 1.2 at a stirring speed of 75 rpm.

#### 2.3.1. Analytical Methods

(1) Surface morphological characterization of porous lactose and quercetin loaded porous lactose by scanning electron microscopy (SEM):

We placed the porous lactose and the quercetin-loaded lactose samples onto carbon tapes on aluminum sample stabs and then used a SS-60-ST Desktop SEM (SHANSHIYIQI, China) with an operating voltage of 15 kV and an operating pressure of 1 Pa to observe the morphologies of the sample after Au-coating for 90 seconds at 15 mA by an CSS-200 Ion Sputter Coater (SHANSHIYIQI, China). Surface morphological characterization of porous lactose and quercetin loaded porous lactose were determined by SEM and we can observe the differences for the porous lactose before and after quercetin loading.

### 2.4. Spectroscopic Characterization

Fourier transform infrared (FTIR) spectroscopy was used to investigate the fingerprint regions for porous lactose and the drug-lactose interactions. It was performed with 64 scans at 400–4000 cm^−1^ in a Nicolet 6700 FTIR spectrometer (Thermo Fisher Scientific). UV-visible spectrophotometer (Cary 60) was used to quantify the drug content.

### 2.5. Differential Scanning Calorimetry (DSC) and X-Ray Diffraction (XRD)

DSC analysis was performed using a HSC-4 DSC (Henven, China). About 10 mg samples used in a sealed pan were measured according to preparation procedure, which was a scanning temperature from room temperature to different temperatures replied on samples, and a ramp rate of 5 °C/min. XRD analysis was useful to investigate crystallinity of the porous lactose and quercetin after being loaded. The samples were loaded into standard plates. The scanning range was 5 ∼30 degree with a scanning rate of 0.02 degree per second, a scanning current of 30 mA, and a scanning voltage of 40 kV.

(2) Pore features of highly-porous lactose before and after quercetin loading:

Using Barrett-Joyner-Halenda (BJH) method to obtain the total pore volume and pore size distribution of porous lactose and using the Brunauer-Emmet-Teller (BET) equations to calculate the total surface area, all samples were carried out at 80^o^C to be outgassed for overnight before the measurements.

## 3. Results and Discussion

### 3.1. Preparation of Porous Lactose

Porous lactose was synthesized by antisolvent method, and the yield was about 70%. As shown in Figure 2(a), the lactose produced is highly porous and similar in size (∼35 microns), while ordinary lactose is almost nonporous [16]. From the enlarged SEM images, porous lactose is composed of aggregated nanocrystals (<1 micron).  Table 1 shows the results of nitrogen physical adsorption. The porous lactose produced has high specific surface area and porosity, with BET surface area of 35.0561 ± 0.4613 m2/g and BJH pore volume of 0.075346 cc/g. High porosity and surface area contribute to higher drug carrying capacity.  Figure 3 (A) shows the pore volume distribution of highly-porous lactose, with typical micropores of about 30 nm and macropores of about 145 nm.

For DSC analysis, the exothermic peak in DSC curve indicates that a part of lactose is amorphous, while the endothermic peak indicates that the substance is crystalline [21, 22].  Figure 5 (A and B) shows DSC curves of porous lactose and *α*-lactose, which indicates that porous lactose and *α*-lactose are crystalline, and the synthesis process of porous lactose does not change its melting peak. The DSC curves of porous lactose and *α*-lactose show a melting peak at 210°C, which is the characteristic peak of crystalline *α*-lactose [23]. The melting peak at 145°C of DSC curve of *α*-lactose monohydrate belongs to its crystallization water, which indicates that the porous lactose produced is anhydrous lactose.

Figure 6 (B) shows the XRD pattern of porous lactose, which also indicates that porous lactose belongs to anhydrous *α*-lactose, and the diffraction lines are located at 19.14, 19.9, 21.6, and 25.6 degrees, which are attributed to anhydrous *α*-lactose [24, 25]. The FTIR fingerprint region (∼1500–500 cm^−1^) can identify lactose. As shown in Figure 4 (A and B), common lactose and porous lactose have a unique peak at 855 cm^−1^, which is the unique peak of *α*-lactose [26].

### 3.2. Crystalline Features, Drug-Loading Capacity, and Release Profile

Quercetin was loaded in lactose by physical adsorption method, and quercetin was adsorbed on the surface of lactose and entered the pores of lactose, so the loading amount of quercetin depends on the surface structure and pore characteristics of lactose [27]. As shown in Table 1, the results of nitrogen physical adsorption study show that porosity and specific surface area decrease, indicating that quercetin deposits in porous lactose nanopores are in crystalline state. In Figures 2(a) and 2(b), compared with the porous lactose before quercetin loading, the SEM photos after quercetin loading have denser and smoother particle surfaces, which is helpful for the deposition of quercetin in lactose.  Figure 3 shows the pore volume distribution of quercetin samples before (A) and after (B) loading. It can be inferred that quercetin molecules have more loading on the pore size from 30 nm to 160 nm, which accounts for a large part of the pore volume. Fourier transform infrared spectra of pure quercetin, *α*-lactose monohydrate, porous lactose, *α*-lactose monohydrate after component loading, and porous lactose particles after component loading are shown in Figure 4. The main characteristic peaks of pure quercetin are at 1100–1600 cm^−1^ and –OH phenol bending (1200–1400 cm^−1^). The main characteristic peak of lactose is at 855 cm^−1^, and these two characteristic peaks appear in quercetin-loaded ordinary lactose and quercetin-loaded porous lactose, which indicates that there is no interaction between quercetin and lactose.

Differential scanning calorimetry has been widely used to effectively determine the physical state of drug molecules [28]. The results of DSC are shown in Figure 5 (E), and quercetin had a melting endotherm at 321 C and also appeared in the DSC curve of quercetin loaded with lactose, indicating that both lactose and lactose-loaded quercetin were crystalline. Figure 6 shows the characteristic diffraction patterns of quercetin at 10.68, 12.42, 15.86, 24.36, 26.52, and 27.24 degrees, indicating that both quercetin and quercetin loaded in lactose are crystalline.  Table 2 shows the loading efficiency of the porous lactose and alpha-lactose. The loading efficiency of quercetin on a porous lactose carrier (20.3% w/w) was higher compared to conventional *α*-lactose (5.2% w/w) which showed significantly lower drug loading due to the good pore characteristics of the porous lactose. The *in vitro* release curve of quercetin from the tablets is shown in Figure 7. The release rate of quercetin in the porous lactose carrier tablet was faster than that of the common *α*-lactose carrier. It was feasible to increase the concentration of quercetin *in vitro* by using porous lactose.

## 4. Conclusions

A novel method was developed in this work to increase the concentration of quercetin *in vitro* using micro-sized highly-porous lactose. In order to improve the poor solubility of hydrophobic drug quercetin and enhance the concentration of its *in vitro* solution, we used the antisolvent method to synthesize high-porosity lactose. The synthesized lactose has good porosity, particle size of ∼35 microns, average pore size of ∼30 nm, BET specific surface area of 35.0561 ± 0.4613°m^2^/g, and BJH pore volume of ∼0.075346 cc/g. After loading of quercetin, the BET specific surface area and BJH pore volume decreased to 28.8735 ± 0.3526°m^2^/g and 0.07315 cc/g, respectively. The DSC curve showed that the porous lactose had a melting peak at 210°C, and the XRD pattern showed diffraction lines at 19.14, 19.9, 21.6, and 25.6 degrees, suggesting that the porous lactose was crystalline *α*-lactose. DSC analysis and XRD analysis of the porous lactose after dosing showed that the quercetin deposits in the nanopores of the porous lactose were in the crystalline state. FTIR spectra showed that there was no interaction between quercetin and lactose. Compared with the common *α*-lactose, quercetin has higher loading efficiency and faster release rate on the porous lactose carrier (20.3% w/w), which is related to the high porosity and high specific surface area of porous lactose.

## Figures and Tables

**Figure 1:** Chemical structure of quercetin.

**Figure 2:** SEM images of the porous lactose particles before (a) and after (b) quercetin loading.

**Figure 3:** Pore volume distribution of the porous lactose before (A) drug loading and after (B) quercetin loading.

**Figure 4:** FTIR spectra of (A) *α*-lactose monohydrate, (B) porous lactose, (C) *α*-lactose monohydrate after quercetin loading, (D) porous lactose particles after quercetin loading, and (E) quercetin.

**Figure 5:** DSC spectra of (A) *α*-lactose monohydrate, (B) porous lactose, (C) quercetin, (D) porous lactose particles after quercetin loading, and (E) *α*-lactose monohydrate after quercetin loading.

**Figure 6:** XRD patterns of (A) *α*-lactose monohydrate, (B) porous lactose, (C) *α*-lactose monohydrate after quercetin loading, (D) porous lactose particles after quercetin loading, and (E) quercetin.

**Figure 7:** Release profiles of quercetin from the porous lactose-carried tablets.

**Table 1:** Pore features of the porous lactose before and after quercetin loading.

	BET surface area (m^2^/g)	BJH pore volume (cc/g)
Porous lactose particles before quercetin loading	35.0561 ± 0.4613	0.075346
Porous lactose particles after quercetin loading	28.8735 ± 0.3526	0.073315

**Table 2:** Loading efficiencies of the porous lactose and *α*-lactose.

	Porous lactose	*α*-lactose
Drug content (%, w/w)		
	20.3	5.2

## Data Availability

The data used to support the findings of this study are included within the article.
